The article "LncRNA TUG1 was upregulated in osteoporosis and regulates the proliferation and apoptosis of osteoclasts" was retracted in 2020. Reason: lack of ethics approval or compliance.

# LncRNA TUG1 was upregulated in osteoporosis and regulates the proliferation and apoptosis of osteoclasts

**DOI:** 10.1186/s13018-019-1430-4

**Published:** 2019-12-09

**Authors:** Ye Han, Chunying Liu, Ming Lei, Shaosong Sun, Wenkui Zheng, Yanan Niu, Xi Xia

**Affiliations:** 1 Department of Orthopaedics, Affiliated Hospital of Hebei University, Baoding City, 071000 Hebei Province People’s Republic of China; 2 Department of Pharmacology, School of Clinical Medicine, Hebei University, Baoding City, 071000 Hebei Province People’s Republic of China; 3 Department of Orthopaedics, Baoding First Central Hospital, No. 320, Great Wall North Street, Baoding City, 071000 Hebei Province People’s Republic of China

**Keywords:** Osteoporosis, lncRNA TUG1, Osteoclast, Proliferation, Apoptosis

## Abstract

**Background:**

Long non-coding RNA (LncRNA) TUG1 plays critical roles in the development of human cancers. Its inhibition has been proved to participate in ankylosing spondylitis, which is an inverse pathological procedure of osteoporosis. In the present study, we aim to investigate the role of lncRNA TUG1 in ankylosing spondylitis.

**Materials and methods:**

Expressions of lncRNA TUG1 in plasma of 98 patients with osteoporosis and 60 healthy participants were detected by real-time quantitative PCR (RT-qPCR). Diagnostic values of lncRNA CASC11 for osteoclasts were performed by the ROC curve with osteoporosis patients as positive and healthy participants as negative. All experiments were repeated 3 times. Mean ± standard deviation was calculated.

**Results:**

We found that plasma lncRNA TUG1 was upregulated in osteoporosis patients than in healthy participants. Upregulation of plasma lncRNA TUG1 distinguished osteoporosis patients from healthy participants. LncRNA TUG1 level increased with the advances of clinical stages. Over-expression of lncRNA TUG1 promoted the proliferation and inhibited the apoptosis of mice osteoclasts, while lncRNA TUG1 siRNA silencing played an opposite role. In addition, lncRNA TUG1 over-expression led to downregulated PTEN, while lncRNA TUG1 siRNA silencing played an opposite role.

**Conclusion:**

Therefore, lncRNA TUG1 is upregulated in osteoporosis and regulates the proliferation and apoptosis of osteoclasts. lncRNA TUG1 knockdown may serve as a promising therapeutic target for osteoporosis by inhibiting the proliferation and promoting the apoptosis of osteoclasts through PTEN.

## Background

Osteoporosis is a bone disease which occurs from the imbalance between bone formation and resorption. The incidence rate of osteoporosis is higher in women than in men. Family history of fracture, low BMI, aging, and smoking are proven to be risk factors for osteoporosis in women [1]. However, a portion of the males, such as the ones with obesity, are also at high risk for osteoporosis [2]. Patients with osteoporosis are usually treated with calcium supplements and hormone replacement [3, 4]. However, therapeutic outcomes are generally unsatisfied due to adverse side effects or poor patient compliance. Therefore, improvement in the treatment of osteoporosis is quite critical.

Long non-coding RNAs (lncRNAs) are a subgroup of non-protein coding RNAs with lengths longer than 200 nucleotides [5]. Growing amounts of literature have shown that lncRNAs are key players in many physiological and pathological processes including osteoporosis [6, 7]. LncRNA taurine upregulated gene 1 (TUG1) has been demonstrated to play an effectual role in the development of human cancers [8, 9]. A recent study showed that the downregulation of lncRNA TUG1 participated in ankylosing spondylitis, which is an inverse pathological change of osteoporosis [10]. This study aimed to analyze the involvement of TUG1 in osteoporosis and to explore its functions. We showed that lncRNA TUG1 was upregulated in osteoporosis and regulated the proliferation and apoptosis of osteoclasts.

## Methods

### Human materials

Blood (5 ml) was extracted from 98 patients with osteoporosis and 60 healthy participants who were admitted to Baoding First Central Hospital from January 2015 to January 2018. Patients with osteoporosis were diagnosed by dual-energy X-ray absorptiometry (T-score of < − 2.5 SD). Blood was used to extract plasma using conventional methods. Inclusion criteria were as follows: (1) patients with osteoclasts who were diagnosed for the first time, (2) patients with complete medical record, and (3) patients who understood the experimental procedure and willing to participate. Exclusion criteria were as follows: (1) patients who were treated 3 months before admission, (2) patients with multiple diseases, and (3) patients who failed to cooperate with researchers. The patient group included 32 males and 66 females, and age range from 30 to 64 years old, with a mean age of 48.2 ± 6.1 years old. Patients were staged according to following methods: stage 1: age at 30 to 35 years old without visible symptoms; stage 2: after age at 35 years old, bone breakdown happens faster than bone buildup, no visible symptoms, only can be detected through bone-density tests; stage 3: age at 45 to 55, bones become so and may break from normal stress; stage 4: bone fractures continue, pain increases, and may cause disability. There were 20 cases at stage I, 28 cases at stage II, 22 cases at stage III, and 28 cases at stage IV. The control group included 22 males and 38 females, and the age range from 30 to 65 years old, with a mean age of 48.7 ± 5.7 years old. No significant differences in age and gender were found between patient and control groups. This study passed the review of Baoding First Central Hospital, and all participants signed informed consent.

### Primary marrow–derived osteoclasts

Bone marrow osteoclast precursors were isolated from C57Bl/6 J mice (8 weeks old, Guangdong Medical Experimental Animal Center, Guangdong, China). Primary marrow–derived osteoclasts were generated from bone marrow osteoclast precursors. All operations here were performed in strict accordance with the methods described by Stiffel et al. [11].

### Real-time quantitative PCR

Total RNA was extracted from plasma using RNAzol® RT RNA Isolation Reagent (Sigma-Aldrich). High-Capacity cDNA Reverse Transcription Kit (Thermo Fisher Scientific) was used to performed reverse transcription. To detect the expression of lncRNA TUG1 and PTEN mRNA, Luna® Universal One-Step RT-qPCR Kit (NEB) was used to prepare PCR reaction systems. Primers of lncRNA TUG1 and β-actin were designed and synthesized by GenePharma (Shanghai, China). The expression of lncRNA TUG1 was normalized to endogenous controls β-actin using the 2^−ΔΔCT^ method.

### Vectors, siRNAs, and cell transfection

Vectors expressing lncRNA TUG1 and empty vectors were designed and constructed by GenePharma (Shanghai, China). LncRNA TUG1 siRNA and scrambled negative control siRNA were also designed and constructed by GenePharma (Shanghai, China). Lipofectamine 2000 reagent (Thermo Fisher Scientific) was used to transfect vectors and siRNAs into primary marrow–derived osteoclasts with vectors at a dose of 10 nM and siRNAs at a dose of 50 nM. Cells only treated with lipofectamine 2000 reagent were control cells. Cells transfected with empty vectors or scrambled negative control siRNA were negative control cells.

### In vitro cell proliferation assay

Expression of lncRNA TUG1 was detected at 24 h after transfection, and cell proliferation was only detected in cases of over-expression rate of lncRNA TUG1 reached 200% and knockdown rate reached 50%. Briefly, primary marrow–derived osteoclasts were harvested and single-cell suspensions were prepared with a cell density of 3 × 10^4^ cells/ml. Cells were transferred to a 96-well plate with 0.1 ml in each well. Cells were cultivated under normal conditions (37 °C, 5% CO_2_), followed by the addition of CCK-8 solution (10ul, Sigma-Aldrich) 24, 48, 72, and 96 h later. Cells were then cultivated for an additional 4 h, and OD values 450 nm were measured to calculate cell proliferation rate.

### Cell apoptosis assay

Expression of lncRNA TUG1 was detected at 24 h after transfection, and cell apoptosis was only detected in cases of over-expression rate of lncRNA TUG1 reached 200% and knockdown rate reached 50%. Briefly, primary marrow–derived osteoclasts were harvested and single-cell suspensions were prepared with a cell density of 3 × 10^4^ cells/ml using serum-free medium. Ten-milliliter cell suspension was added into each well of a 6-well plate, and 0.25% trypsin digestion was performed. After cells were cultivated for 48 h, staining with Annexin V-FITC (Dojindo, Japan) and propidium iodide (PI) was performed and cell apoptosis was detected by flow cytometry.

### Statistical analysis

All experiments were repeated 3 times, and the mean ± standard deviation was calculated. The unpaired *t* test was used for comparisons between 2 groups, and one-way ANOVA followed by Tukey’s test was performed to compare 3 groups. Diagnostic values of lncRNA CASC11 for osteoclasts were performed by the receiver operating characteristic (ROC) curve with osteoporosis patients as true positive cases and healthy participants as true negative cases. Differences with *p* < 0.05 were statistically significant.

## Results

### Plasma lncRNA TUG1 was upregulated in osteoporosis patients than in healthy participants

Expression of lncRNA TUG1 in plasma of 98 patients with osteoporosis and 60 healthy participants was detected by RT-qPCR. Compared with healthy participants, plasma levels of lncRNA TUG1 were significantly higher in osteoporosis patients (Fig. 1, *p* < 0.05).

**Fig. 1:** Plasma lncRNA TUG1 was upregulated in osteoporosis patients than in healthy participants. RT-qPCR results showed that plasma levels of lncRNA TUG1 were significantly higher in osteoporosis patients than in healthy participants (*p < 0.05)

### Upregulation of plasma lncRNA TUG1 distinguished osteoporosis patients from healthy participants

Diagnostic values of lncRNA CASC11 for osteoclasts were performed by the ROC curve with osteoporosis patients as true positive cases and healthy participants as true negative cases. As shown in Fig. 2, the area under the curve was 0.90, with a standard error of 0.023 and a 95% confidence interval of 0.86–0.95. ROC curve analysis showed that the upregulation of plasma lncRNA TUG1 distinguished osteoporosis patients from healthy participants.

**Fig. 2:** Upregulation of plasma lncRNA TUG1 distinguished osteoporosis patients from healthy participants

### Plasma lncRNA TUG1 level increased with increase in stages

Among 98 patients with osteoporosis, there were 20 cases at stage I, 28 cases at stage II, 22 cases at stage III, and 28 cases at stage IV. As shown in Fig. 3, plasma levels of lncRNA TUG1 were significantly increased with an increase in stages (*p* < 0.05).

**Fig. 3:** Plasma lncRNA TUG1 level increased with increase in stages. Plasma levels of lncRNA TUG1 significantly increased with an increase in stages (*p < 0.05)

### LcRNA TUG1 regulates proliferation and apoptosis of mice osteoclasts

Over-expression and siRNA silencing experiments were performed to investigate the role of lncRNA TUG1 in the regulation of the proliferation and apoptosis of mice osteoclasts. Compared with control and negative control groups, over-expression of lncRNA TUG1 significantly promoted the proliferation (Fig. 4a, *p* < 0.05) and inhibited the apoptosis (Fig. 4b, *p* < 0.05) of mice osteoclasts. In addition, lncRNA TUG1 siRNA silencing played the opposite role. Moreover, lncRNA TUG1 over-expression led to downregulated PTEN mRNA, while lncRNA TUG1 siRNA silencing played an opposite role (Fig. 4c, *p* < 0.05).

**Fig. 4:** LcRNA TUG1 regulates proliferation and apoptosis of mice osteoclasts. Over-expression of lncRNA TUG1 significantly promoted the proliferation (**a**) and inhibited the apoptosis (**b**) of mice osteoclasts, while lncRNA TUG1 siRNA silencing played an opposite role. Moreover, lncRNA TUG1 over-expression led to downregulated PTEN mRNA, while lncRNA TUG1 siRNA silencing played an opposite role (**c**), (*p < 0.05)

## Discussion

LncRNA TUG1 inhibition participates in ankylosing spondylitis, which is an inverse pathological change of osteoporosis [10], indicating the potential involvement of lncRNA TUG1 in osteoporosis. The key finding of the present study is that lncRNA TUG1 is upregulated in osteoporosis and lncRNA TUG1 may regulate the proliferation and apoptosis of osteoporosis.

The development and progression of osteoporosis are accompanied by changes in the expression pattern of a large set of lncRNAs [7], indicating the involvement of lncRNAs in this disease. However, most studies focused on the functions of lncRNAs in postmenopausal osteoporosis, which is related to hormone levels [12, 13]. Studies on the roles of lncRNAs in general osteoporosis are rare. In a recent study, Zhang et al. reported that lncRNA MSC-AS1 can alleviate osteoporosis by promoting osteogenic differentiation through the upregulation of BMP2 by sponging miR-140-5p [14]. In another study, Zheng et al. showed that lncRNA MALAT1 could inhibit mesenchymal stem cell osteogenic differentiation of rat osteoporosis model [15]. LncRNA TUG1 plays the role of oncogene or tumor suppressor gene in different types of human cancers [8, 16]. A recent study showed that lncRNA TUG1 expression was inhibited in ankylosing spondylitis [10]. In the present study, we first showed the upregulated expression pattern of lncRNA TUG1 in osteoporosis than in ankylosing spondylitis people, further confirming the inverse pathological change of osteoporosis to ankylosing spondylitis. In effect, upregulation of plasma lncRNA TUG1 distinguished osteoporosis patients from healthy participants. Therefore, plasma lncRNA TUG1 may serve as a potential diagnostic marker for osteoporosis.

Osteoclasts play a key role in bone resorption [17], which is usually accelerated in patients with osteoporosis [18]. Therefore, inhibition of the proliferation of osteoclasts is considered as a promising therapeutic target for the treatment of osteoporosis [19, 20]. It is known that the proliferation of osteoclasts can be regulated by lncRNAs [21]. Phosphatase and tensin homolog (PTEN) signaling has critical roles in the apoptosis of osteoclasts [22]. In the present study, we showed that lncRNA TUG1 positively regulated the proliferation of osteoclasts and negatively regulated the apoptosis of osteoclasts through PTEN. Therefore, inhibition of lncRNA TUG1 may serve as a promising therapeutic target for osteoporosis. However, more experimental and clinical studies are needed to further confirm our conclusions.

Our study did not elucidate the mechanism of the actions of lncRNA TUG1 in regulating the proliferation and apoptosis of osteoclasts. However, it is known that TUG1 can sponge miR-204-5p to promote osteoblast differentiation [23]. It has been established that many signaling pathways, including Runt-related transcription factors, play critical roles in osteoblast proliferation and differentiation [24, 25]. Our future studies will try to characterize the potential interactions between lncRNA TUG1 and these pathways.

## Conclusion

In conclusion, lncRNA TUG1 was upregulated in osteoporosis and lncRNA TUG1 knockdown may serve as a promising therapeutic target for osteoporosis by inhibiting the proliferation and promoting the apoptosis of osteoclasts.

## Data Availability

The analyzed data sets generated during the study are available from the corresponding author on reasonable request.

## Abbreviation

LncRNA: Long non-coding RNA
RT-qPCR: Real-time quantitative PCR
ROC: Receiver operating characteristic
